The article "Diaqua-1κO,3κO-di-μ-cyanido-1:2κ2 N:C;2:3κ2 C:N-dicyanido-2κ2 C-bis­{4,4′-dibromo-2,2′-[propane-1,2-diylbis(nitrilo­methyl­idyne)]diphenolato}-1κ4 O,N,N′,O′;3κ4 O,N,N′,O′-1,3-di­iron(III)-2-nickel(II)" was retracted in 2011. Reasons: fabricated or falsified data; errors in the data.

# Diaqua-1κ*O*,3κ*O*-di-μ-cyanido-1:2κ^2^ *N*:*C*;2:3κ^2^ *C*:*N*-dicyanido-2κ^2^ *C*-bis­{4,4′-dibromo-2,2′-[propane-1,2-diylbis(nitrilo­methyl­idyne)]diphenolato}-1κ^4^ *O*,*N*,*N*′,*O*′;3κ^4^ *O*,*N*,*N*′,*O*′-1,3-di­iron(III)-2-nickel(II)

**DOI:** 10.1107/S1600536808017893

**Published:** 2008-06-19

**Authors:** Xiutang Zhang, Peihai Wei, Bin Li

**Affiliations:** a Department of Chemistry and Chemical Engineering, ShanDong Institute of Education, Jinan 250013, People’s Republic of China

## Abstract

The title compound, [Fe_2_Ni(C_17_H_14_Br_2_N_2_O_2_)_2_(CN)_4_(H_2_O)_2_] or [{Fe(C_17_H_14_Br_2_N_2_O_2_)(H_2_O)}_2_(μ-CN)_2_{Ni(CN)_2_}], is iso­structural with its Mn^III^-containing analogue. Each Fe^III^ atom is chelated by a Schiff base ligand *via* two N and two O atoms and is additionally coordinated by a water mol­ecule, forming a slightly distorted octa­hedral geometry. The two Fe^III^ centres are bridged by a square-planar Ni(CN)_4_ unit, which lies on an inversion centre. A two-dimensional network is formed *via* O—H⋯O and O—H⋯N hydrogen bonds.

## Related literature

For related literature, see: Kuang *et al.* (2002 ▶); Kuchar *et al.* (2003 ▶); Yang *et al.* (2003 ▶). For the isostructural Mn^III^-containing compound, see: Sun *et al.* (2008 ▶).

## Experimental

### 

#### Crystal data

[Fe_2_Ni(C_17_H_14_Br_2_N_2_O_2_)_2_(CN)_4_(H_2_O)_2_]
*M* *_r_* = 1186.71
Monoclinic,
*a* = 11.599 (2) Å
*b* = 13.538 (3) Å
*c* = 14.715 (3) Å
β = 112.04 (3)°
*V* = 2141.8 (7) Å^3^
*Z* = 2
Mo *K*α radiation
μ = 4.89 mm^−1^
*T* = 293 (2) K
0.10 × 0.10 × 0.10 mm

#### Data collection

Bruker APEXII CCD diffractometer
Absorption correction: multi-scan (*SADABS*; Bruker, 2001 ▶) *T*_min_ = 0.449, *T*_max_ = 0.641
13404 measured reflections
3699 independent reflections
2263 reflections with *I* > 2σ(*I*)
*R*_int_ = 0.085

#### Refinement

*R*[*F* ^2^ > 2σ(*F* ^2^)] = 0.066
*wR*(*F* ^2^) = 0.181
*S* = 1.00
3699 reflections
276 parameters
3 restraints
H atoms treated by a mixture of independent and constrained refinement
Δρ_max_ = 0.96 e Å^−3^
Δρ_min_ = −0.64 e Å^−3^

### 

Data collection: *APEX2* (Bruker, 2004 ▶); cell refinement: *SAINT-Plus* (Bruker, 2001 ▶); data reduction: *SAINT-Plus*; program(s) used to solve structure: *SHELXS97* (Sheldrick, 2008 ▶); program(s) used to refine structure: *SHELXL97* (Sheldrick, 2008 ▶); molecular graphics: *SHELXTL* (Sheldrick, 2008 ▶); software used to prepare material for publication: *SHELXTL*).

## Supplementary Material

Crystal structure: contains datablocks global, I. DOI: 10.1107/S1600536808017893/cf2205sup1.cif

Structure factors: contains datablocks I. DOI: 10.1107/S1600536808017893/cf2205Isup2.hkl

Additional supplementary materials:  crystallographic information; 3D view; checkCIF report

The article "Diaqua-1κO,3κO-di-μ-cyanido-1:2κ2 N:C;2:3κ2 C:N-dicyanido-2κ2 C-bis­{4,4′-dibromo-2,2′-[propane-1,2-diylbis(nitrilo­methyl­idyne)]diphenolato}-1κ4 O,N,N′,O′;3κ4 O,N,N′,O′-1,3-di­iron(III)-2-nickel(II)" was retracted in 2011. Reasons: fabricated or falsified data; errors in the data.

## Figures and Tables

**Table 1:** Hydrogen-bond geometry (Å, °)

*D*—H⋯*A*	*D*—H	H⋯*A*	*D*⋯*A*	*D*—H⋯*A*
O3—H1*W*⋯O1^i^	0.81 (2)	2.09 (4)	2.859 (7)	159 (8)
O3—H2*W*⋯N2^ii^	0.81 (2)	2.02 (2)	2.813 (9)	167 (7)

Symmetry codes: (i) ; (ii) .

## supplementary crystallographic information

### Comment

Cyanide-bridged oligonuclear complexes with chain-like arrangements of metal ions and cyanide ligands have been studied for a long time due to the good electronic conductivity between the metallic groups (Kuang *et al.*, 2002; Kuchar *et al.*, 2003; Yang *et al.*, 2003). In this context, bulk properties such as magnetism, luminescence, electrical conductivity resulting from metal-metal charge transfer like multi-redox steps, mixed valence and long-range electronic interactions prompted us to report our research work on cyanide-bridged complexes. In this paper, we report the structure of the title compound, (I).  It is isostructural with its Mn^III^-containing analogue (Sun *et al.*, 2008).

As shown in Fig. 1, each Fe^III^ atom is chelated by a Schiff base ligand *via* two N and two O atoms and is additionally coordinated by a water molecule, forming a slightly distorted octahedral geometry. The Schiff base lies in the equatorial plane, and the cyanido and aqua ligands lie in the axial coordination sites. The Fe—N and Fe—O axial bond lengths are much longer than the equatorial ones. A centrosymmetric square-planar Ni(CN)_4_ unit links two Fe^III^ centres. With O—H···O and O—H···N hydrogen bonds, a two-dimensional network is formed, as shown in Fig. 2.

### Experimental

A mixture of iron(III) acetylacetonate (1 mmol), *N*,*N*'-bis(2-hydroxy-5-bromobenzyl)-1,2-diaminopropane (1 mmol), and dipotassium tetracyanidonickelate(II) (1 mmol) in 20 ml methanol was refluxed for several hours. The cooled solution was filtered and the filtrate was kept in an ice box. One week later, brown blocks of (I) were obtained with a yield of 5%. Anal. Calc. for C_38_H_32_Br_4_Fe_2_N_8_NiO_6_: C 38.43, H 2.70, N 9.44%; Found: C 38.40, H 2.63, N 9.39.

### Refinement

All C-bound H atoms were placed in calculated positions with C—H = 0.93 Å and refined as riding with *U*_iso_(H) = 1.2*U*_eq_(C). H atoms on the aqua ligand were located in a difference density map and were refined with the distance restraint O—H = 0.82 (1) Å.

### Crystal data

**Table:**

[Fe_2_Ni(C_17_H_14_Br_2_N_2_O_2_)_2_(CN)_4_(H_2_O)_2_]	*F*_000_ = 1168
*M**_r_* = 1186.71	*D*_x_ = 1.840 Mg m^−^^3^
Monoclinic, *P*2_1_/*n*	Mo *K*α radiation λ = 0.71073 Å
Hall symbol: -P 2yn	Cell parameters from 3699 reflections
*a* = 11.599 (2) Å	θ = 3.0–25.1º
*b* = 13.538 (3) Å	µ = 4.89 mm^−^^1^
*c* = 14.715 (3) Å	*T* = 293 (2) K
β = 112.04 (3)º	Block, brown
*V* = 2141.8 (7) Å^3^	0.10 × 0.10 × 0.10 mm
*Z* = 2	

The article "Diaqua-1κO,3κO-di-μ-cyanido-1:2κ2 N:C;2:3κ2 C:N-dicyanido-2κ2 C-bis­{4,4′-dibromo-2,2′-[propane-1,2-diylbis(nitrilo­methyl­idyne)]diphenolato}-1κ4 O,N,N′,O′;3κ4 O,N,N′,O′-1,3-di­iron(III)-2-nickel(II)" was retracted in 2011. Reasons: fabricated or falsified data; errors in the data.

### Data collection

**Table:**

Bruker APEXII CCD diffractometer	3699 independent reflections
Radiation source: fine-focus sealed tube	2263 reflections with *I* > 2σ(*I*)
Monochromator: graphite	*R*_int_ = 0.085
*T* = 293(2) K	θ_max_ = 25.1º
φ and ω scans	θ_min_ = 3.0º
Absorption correction: multi-scan(SADABS; Bruker, 2001)	*h* = −13→12
*T*_min_ = 0.449, *T*_max_ = 0.641	*k* = −16→15
13404 measured reflections	*l* = −17→17

### Refinement

**Table:**

Refinement on *F*^2^	Secondary atom site location: difference Fourier map
Least-squares matrix: full	Hydrogen site location: inferred from neighbouring sites
*R*[*F*^2^ > 2σ(*F*^2^)] = 0.066	H atoms treated by a mixture of independent and constrained refinement
*wR*(*F*^2^) = 0.181	*w* = 1/[σ^2^(*F*_o_^2^) + (0.09*P*)^2^] where *P* = (*F*_o_^2^ + 2*F*_c_^2^)/3
*S* = 1.00	(Δ/σ)_max_ < 0.001
3699 reflections	Δρ_max_ = 0.96 e Å^−^^3^
276 parameters	Δρ_min_ = −0.64 e Å^−^^3^
3 restraints	Extinction correction: none
Primary atom site location: structure-invariant direct methods	

### Special details

**Table:**

Geometry. All e.s.d.'s (except the e.s.d. in the dihedral angle between two l.s. planes) are estimated using the full covariance matrix. The cell e.s.d.'s are taken into account individually in the estimation of e.s.d.'s in distances, angles and torsion angles; correlations between e.s.d.'s in cell parameters are only used when they are defined by crystal symmetry. An approximate (isotropic) treatment of cell e.s.d.'s is used for estimating e.s.d.'s involving l.s. planes.
Refinement. Refinement of *F*^2^ against ALL reflections. The weighted *R*-factor *wR* and goodness of fit *S* are based on *F*^2^, conventional *R*-factors *R* are based on *F*, with *F* set to zero for negative *F*^2^. The threshold expression of *F*^2^ > σ(*F*^2^) is used only for calculating *R*-factors(gt) *etc*. and is not relevant to the choice of reflections for refinement. *R*-factors based on *F*^2^ are statistically about twice as large as those based on *F*, and *R*- factors based on ALL data will be even larger.

### Fractional atomic coordinates and isotropic or equivalent isotropic displacement parameters (Å^2^)

**Table:**

	*x*	*y*	*z*	*U*_iso_*/*U*_eq_	
Fe1	0.29547 (11)	0.95323 (8)	0.36728 (8)	0.0341 (4)	
Ni1	0.0000	1.0000	0.0000	0.0334 (4)	
Br1	−0.07330 (10)	1.37221 (7)	0.43825 (7)	0.0569 (4)	
Br2	0.75936 (10)	0.61244 (8)	0.30711 (8)	0.0621 (4)	
C1	0.1210 (8)	0.9936 (5)	0.1261 (6)	0.035 (2)	
C2	−0.0637 (8)	0.8804 (6)	0.0276 (6)	0.037 (2)	
C3	0.2234 (8)	1.1459 (6)	0.4134 (6)	0.034 (2)	
C4	0.2476 (8)	1.2492 (5)	0.4247 (5)	0.033 (2)	
H4	0.3242	1.2728	0.4277	0.039*	
C5	0.1608 (9)	1.3146 (6)	0.4311 (6)	0.042 (2)	
H5	0.1780	1.3819	0.4362	0.050*	
C6	0.0471 (9)	1.2807 (6)	0.4303 (6)	0.042 (2)	
C7	0.0185 (9)	1.1818 (6)	0.4197 (6)	0.045 (2)	
H7	−0.0581	1.1603	0.4187	0.054*	
C8	0.1029 (8)	1.1136 (5)	0.4104 (6)	0.037 (2)	
C9	0.0680 (8)	1.0105 (6)	0.3966 (6)	0.035 (2)	
H9	−0.0079	0.9939	0.4004	0.042*	
C10	0.0874 (10)	0.8350 (7)	0.3700 (9)	0.067 (3)	
H10A	0.1154	0.8044	0.4343	0.080*	
H10B	−0.0028	0.8331	0.3424	0.080*	
C11	0.1355 (9)	0.7815 (7)	0.3082 (9)	0.067 (3)	
H11	0.0893	0.8088	0.2429	0.080*	
C12	0.1048 (10)	0.6739 (6)	0.2961 (8)	0.060 (3)	
H12A	0.1567	0.6390	0.3537	0.091*	
H12B	0.1188	0.6491	0.2400	0.091*	
H12C	0.0191	0.6646	0.2869	0.091*	
C13	0.3443 (8)	0.7546 (5)	0.3198 (5)	0.032 (2)	
H13	0.3196	0.6893	0.3047	0.039*	
C14	0.4688 (8)	0.7786 (6)	0.3302 (5)	0.033 (2)	
C15	0.5437 (9)	0.7030 (6)	0.3193 (5)	0.038 (2)	
H15	0.5141	0.6384	0.3116	0.046*	
C16	0.6591 (9)	0.7209 (7)	0.3197 (6)	0.049 (3)	
C17	0.7053 (9)	0.8158 (7)	0.3289 (6)	0.048 (2)	
H17	0.7829	0.8280	0.3262	0.058*	
C18	0.6337 (8)	0.8932 (6)	0.3422 (6)	0.039 (2)	
H18	0.6657	0.9570	0.3509	0.047*	
C19	0.5155 (8)	0.8770 (6)	0.3428 (5)	0.033 (2)	
N1	0.1906 (7)	0.9903 (4)	0.2063 (5)	0.0368 (18)	
N2	−0.0938 (7)	0.8039 (5)	0.0441 (5)	0.046 (2)	
N3	0.1306 (6)	0.9396 (5)	0.3796 (5)	0.0400 (18)	
N4	0.2649 (6)	0.8131 (4)	0.3289 (4)	0.0294 (16)	
O1	0.4524 (5)	0.9530 (3)	0.3561 (4)	0.0309 (13)	
O2	0.3095 (5)	1.0870 (4)	0.4047 (4)	0.0308 (13)	
O3	0.3783 (5)	0.9024 (4)	0.5250 (4)	0.0352 (14)	
H1W	0.433 (5)	0.942 (3)	0.547 (6)	0.042*	
H2W	0.397 (6)	0.8444 (16)	0.530 (6)	0.042*	

The article "Diaqua-1κO,3κO-di-μ-cyanido-1:2κ2 N:C;2:3κ2 C:N-dicyanido-2κ2 C-bis­{4,4′-dibromo-2,2′-[propane-1,2-diylbis(nitrilo­methyl­idyne)]diphenolato}-1κ4 O,N,N′,O′;3κ4 O,N,N′,O′-1,3-di­iron(III)-2-nickel(II)" was retracted in 2011. Reasons: fabricated or falsified data; errors in the data.

### Atomic displacement parameters (Å^2^)

**Table:**

	*U*^11^	*U*^22^	*U*^33^	*U*^12^	*U*^13^	*U*^23^
Fe1	0.0365 (8)	0.0271 (7)	0.0247 (6)	0.0005 (5)	−0.0045 (5)	−0.0009 (5)
Ni1	0.0368 (9)	0.0254 (8)	0.0201 (7)	−0.0002 (6)	−0.0101 (6)	0.0006 (6)
Br1	0.0723 (8)	0.0473 (6)	0.0454 (6)	0.0242 (5)	0.0155 (5)	−0.0023 (5)
Br2	0.0537 (7)	0.0690 (8)	0.0549 (7)	0.0211 (5)	0.0105 (5)	−0.0137 (5)
C1	0.054 (6)	0.012 (4)	0.029 (5)	−0.002 (4)	0.003 (4)	0.000 (3)
C2	0.036 (5)	0.032 (5)	0.024 (4)	0.002 (4)	−0.010 (4)	0.000 (4)
C3	0.037 (5)	0.029 (4)	0.022 (4)	0.004 (4)	−0.007 (4)	−0.003 (3)
C4	0.039 (5)	0.031 (4)	0.018 (4)	−0.008 (4)	−0.001 (4)	0.001 (3)
C5	0.060 (7)	0.028 (5)	0.031 (5)	0.011 (5)	0.010 (5)	−0.004 (4)
C6	0.056 (6)	0.026 (5)	0.032 (5)	0.006 (4)	0.005 (4)	0.001 (4)
C7	0.052 (6)	0.054 (6)	0.022 (4)	0.011 (5)	0.005 (4)	−0.006 (4)
C8	0.044 (6)	0.030 (5)	0.024 (4)	0.009 (4)	−0.002 (4)	0.001 (3)
C9	0.031 (5)	0.038 (5)	0.030 (4)	0.001 (4)	0.004 (4)	−0.004 (4)
C10	0.064 (7)	0.043 (6)	0.104 (9)	−0.016 (5)	0.045 (7)	−0.025 (6)
C11	0.047 (7)	0.040 (6)	0.112 (10)	−0.004 (5)	0.030 (7)	−0.028 (6)
C12	0.059 (7)	0.039 (5)	0.076 (8)	−0.008 (5)	0.017 (6)	−0.008 (5)
C13	0.040 (5)	0.019 (4)	0.027 (4)	0.000 (4)	−0.001 (4)	−0.001 (3)
C14	0.034 (5)	0.034 (5)	0.020 (4)	0.009 (4)	−0.003 (4)	−0.008 (3)
C15	0.047 (6)	0.038 (5)	0.019 (4)	0.001 (4)	−0.001 (4)	0.000 (3)
C16	0.053 (6)	0.052 (6)	0.025 (5)	0.020 (5)	−0.004 (4)	−0.009 (4)
C17	0.043 (6)	0.054 (6)	0.043 (6)	−0.001 (5)	0.013 (5)	−0.011 (5)
C18	0.042 (6)	0.045 (5)	0.025 (4)	−0.003 (4)	0.006 (4)	−0.004 (4)
C19	0.035 (5)	0.043 (5)	0.010 (4)	0.010 (4)	−0.005 (3)	−0.003 (3)
N1	0.042 (4)	0.026 (4)	0.024 (4)	−0.007 (3)	−0.009 (3)	0.000 (3)
N2	0.055 (5)	0.029 (4)	0.037 (4)	−0.008 (4)	−0.001 (4)	−0.005 (3)
N3	0.038 (4)	0.033 (4)	0.043 (4)	−0.003 (3)	0.007 (4)	−0.011 (3)
N4	0.028 (4)	0.026 (4)	0.026 (4)	0.000 (3)	0.000 (3)	−0.001 (3)
O1	0.031 (3)	0.028 (3)	0.023 (3)	0.002 (2)	−0.001 (2)	0.001 (2)
O2	0.031 (3)	0.028 (3)	0.025 (3)	0.001 (2)	0.001 (2)	0.001 (2)
O3	0.040 (4)	0.025 (3)	0.025 (3)	−0.004 (3)	−0.004 (3)	−0.003 (3)

The article "Diaqua-1κO,3κO-di-μ-cyanido-1:2κ2 N:C;2:3κ2 C:N-dicyanido-2κ2 C-bis­{4,4′-dibromo-2,2′-[propane-1,2-diylbis(nitrilo­methyl­idyne)]diphenolato}-1κ4 O,N,N′,O′;3κ4 O,N,N′,O′-1,3-di­iron(III)-2-nickel(II)" was retracted in 2011. Reasons: fabricated or falsified data; errors in the data.

### Geometric parameters (Å, °)

**Table:**

Fe1—O2	1.882 (5)	C9—H9	0.930
Fe1—O1	1.888 (6)	C10—C11	1.430 (13)
Fe1—N4	1.973 (6)	C10—N3	1.490 (11)
Fe1—N3	1.996 (7)	C10—H10A	0.970
Fe1—O3	2.261 (5)	C10—H10B	0.970
Fe1—N1	2.276 (6)	C11—N4	1.478 (11)
Ni1—C1^i^	1.862 (8)	C11—C12	1.494 (11)
Ni1—C1	1.862 (8)	C11—H11	0.980
Ni1—C2	1.886 (9)	C12—H12A	0.960
Ni1—C2^i^	1.886 (9)	C12—H12B	0.960
Br1—C6	1.903 (9)	C12—H12C	0.960
Br2—C16	1.924 (9)	C13—N4	1.260 (9)
C1—N1	1.154 (10)	C13—C14	1.431 (11)
C2—N2	1.148 (9)	C13—H13	0.930
C3—O2	1.322 (9)	C14—C15	1.390 (11)
C3—C4	1.423 (10)	C14—C19	1.424 (11)
C3—C8	1.449 (12)	C15—C16	1.359 (13)
C4—C5	1.371 (11)	C15—H15	0.930
C4—H4	0.930	C16—C17	1.378 (12)
C5—C6	1.393 (13)	C17—C18	1.396 (12)
C5—H5	0.930	C17—H17	0.930
C6—C7	1.374 (11)	C18—C19	1.392 (12)
C7—C8	1.389 (12)	C18—H18	0.930
C7—H7	0.930	C19—O1	1.318 (9)
C8—C9	1.445 (10)	O3—H1W	0.80 (6)
C9—N3	1.284 (10)	O3—H2W	0.81 (2)
			
O2—Fe1—O1	92.7 (2)	N3—C10—H10B	109.6
O2—Fe1—N4	174.5 (3)	H10A—C10—H10B	108.2
O1—Fe1—N4	92.8 (3)	C10—C11—N4	109.3 (8)
O2—Fe1—N3	92.5 (2)	C10—C11—C12	115.9 (10)
O1—Fe1—N3	174.6 (2)	N4—C11—C12	119.0 (8)
N4—Fe1—N3	82.0 (3)	C10—C11—H11	103.5
O2—Fe1—O3	92.1 (2)	N4—C11—H11	103.5
O1—Fe1—O3	92.1 (2)	C12—C11—H11	103.5
N4—Fe1—O3	87.8 (2)	C11—C12—H12A	109.5
N3—Fe1—O3	86.1 (3)	C11—C12—H12B	109.5
O2—Fe1—N1	92.7 (2)	H12A—C12—H12B	109.5
O1—Fe1—N1	93.8 (2)	C11—C12—H12C	109.5
N4—Fe1—N1	86.9 (2)	H12A—C12—H12C	109.5
N3—Fe1—N1	87.6 (3)	H12B—C12—H12C	109.5
O3—Fe1—N1	172.3 (2)	N4—C13—C14	126.5 (7)
C1^i^—Ni1—C1	180.0 (4)	N4—C13—H13	116.8
C1^i^—Ni1—C2	92.6 (3)	C14—C13—H13	116.8
C1—Ni1—C2	87.4 (3)	C15—C14—C19	118.8 (8)
C1^i^—Ni1—C2^i^	87.4 (3)	C15—C14—C13	118.0 (7)
C1—Ni1—C2^i^	92.6 (3)	C19—C14—C13	123.0 (7)
C2—Ni1—C2^i^	180.000 (1)	C16—C15—C14	121.7 (8)
N1—C1—Ni1	176.0 (9)	C16—C15—H15	119.2
N2—C2—Ni1	174.3 (8)	C14—C15—H15	119.2
O2—C3—C4	118.7 (8)	C15—C16—C17	120.9 (9)
O2—C3—C8	124.7 (7)	C15—C16—Br2	119.5 (7)
C4—C3—C8	116.5 (7)	C17—C16—Br2	119.6 (8)
C5—C4—C3	121.7 (8)	C16—C17—C18	118.9 (9)
C5—C4—H4	119.2	C16—C17—H17	120.5
C3—C4—H4	119.2	C18—C17—H17	120.5
C4—C5—C6	120.3 (8)	C19—C18—C17	121.5 (8)
C4—C5—H5	119.9	C19—C18—H18	119.2
C6—C5—H5	119.9	C17—C18—H18	119.2
C7—C6—C5	120.6 (8)	O1—C19—C18	118.8 (8)
C7—C6—Br1	119.4 (7)	O1—C19—C14	123.0 (8)
C5—C6—Br1	119.9 (6)	C18—C19—C14	118.2 (8)
C6—C7—C8	120.7 (9)	C1—N1—Fe1	165.6 (7)
C6—C7—H7	119.7	C9—N3—C10	122.3 (8)
C8—C7—H7	119.7	C9—N3—Fe1	125.4 (6)
C7—C8—C9	119.0 (9)	C10—N3—Fe1	112.3 (6)
C7—C8—C3	120.2 (8)	C13—N4—C11	121.5 (7)
C9—C8—C3	120.8 (7)	C13—N4—Fe1	125.1 (6)
N3—C9—C8	126.9 (8)	C11—N4—Fe1	113.4 (5)
N3—C9—H9	116.6	C19—O1—Fe1	128.4 (5)
C8—C9—H9	116.6	C3—O2—Fe1	128.5 (5)
C11—C10—N3	110.1 (8)	Fe1—O3—H1W	100 (6)
C11—C10—H10A	109.6	Fe1—O3—H2W	112 (6)
N3—C10—H10A	109.6	H1W—O3—H2W	118 (4)
C11—C10—H10B	109.6		

Symmetry codes: (i) −*x*, −*y*+2, −*z*.

The article "Diaqua-1κO,3κO-di-μ-cyanido-1:2κ2 N:C;2:3κ2 C:N-dicyanido-2κ2 C-bis­{4,4′-dibromo-2,2′-[propane-1,2-diylbis(nitrilo­methyl­idyne)]diphenolato}-1κ4 O,N,N′,O′;3κ4 O,N,N′,O′-1,3-di­iron(III)-2-nickel(II)" was retracted in 2011. Reasons: fabricated or falsified data; errors in the data.

### Hydrogen-bond geometry (Å, °)

**Table:**

*D*—H···*A*	*D*—H	H···*A*	*D*···*A*	*D*—H···*A*
O3—H1W···O1^ii^	0.81 (2)	2.09 (4)	2.859 (7)	159 (8)
O3—H2W···N2^iii^	0.81 (2)	2.02 (2)	2.813 (9)	167 (7)

Symmetry codes: (ii) −*x*+1, −*y*+2, −*z*+1; (iii) *x*+1/2, −*y*+3/2, *z*+1/2.
